# BCYRN1 is correlated with progression and prognosis in gastric cancer

**DOI:** 10.1042/BSR20190505

**Published:** 2019-11-15

**Authors:** Hongbing Zhai, Yanju Li

**Affiliations:** 1 Department of Gastroenterology, Xianyang Central Hospital, Xianyang 712000, Shaanxi, China; 2 Department of Pathology, Yanan University Affiliated Hospital, Yan’an 716000, Shaanxi, China

**Keywords:** BCYRN1, biomarkers, gastric cancer, large intervening non-coding RNA

## Abstract

Long non-coding RNA brain cytoplasmic RNA 1 (BCYRN1) has been found to play an important role in tumorigenesis of a variety of tumors including gastric cancer (GC). However, the prognostic significance and molecular mechanism of BCYRN1 was still unknown in GC. In the present study, we found BCYRN1 expression was dramatically elevated in GC tissues and cell lines, and positively associated with tumor depth, lymph node metastasis and clinical stage in patients with GC. Moreover, univariate and multivariate Cox regression analyses demonstrated that high BCYRN1 expression was independent prognostic factor for overall survival in GC patients. In lncRNA-microRNA interactome database, we found that there were putative binding sites between BCYRN1 and miR-204-5p. Furthermore, we confirmed that down-regulation of BCYRN1 inhibited GC cell proliferation, migration and invasion through directly up-regulated miR-204-5p expression. In conclusion, BCYRN1 acts as a promising prognostic predictor in GC patients and regulated GC cell proliferation, cell cycle, migration and invasion through targeting miR-204-5p.

## Introduction

Gastric cancer (GC) is the fourth prevalent cancer and the second leading cause of cancer deaths worldwide [1]. Although a decreasing incidence of GC was observed in many countries due to the changes in eating habits and environment, GC remains prevalent in East Asia, especially in China, Japan and Korea [2]. Despite some advances in the diagnosis and treatment, the GC patients’ clinical outcome has not improved significantly at present [3]. In most countries, the 5-year overall survival rate for GC patients remains below 20% [4]. Therefore, the identification of mechanism of GC tumorigenesis can provide new insight to develop targeted therapy and improve the prognosis of GC patients.

Long non-coding RNA brain cytoplasmic RNA 1 (BCYRN1), also known as BC200 RNA, is a 200-nucleotide non-coding RNA transcribed from human chromosome 2p21 between *CALM2* and *EPCAM* genes [5,6]. Originally, BCYRN1 was identified as a brain-specific non-coding RNA involved in neurodegenerative disease [7]. Subsequently, BCYRN1 was found to function as an oncogenic lncRNA in several types of human tumor [8]. In GC, BCYRN1 was increased in GC, and associated with TNM stage and tumor size [9]. In addition, BCYRN1 promoted GC cell proliferation, migration and invasion *in vitro* [9]. However, the prognostic significance and molecular mechanism of BCYRN1 were still unknown in GC. Thus, we further explored the clinical and prognostic significance of BCYRN1 in GC patients through analyzing the correlation between BCYRN1 expression and clinicopathologic features including overall survival. Moreover, we analyzed lncRNA-microRNA interactome database and found that there were putative binding sites between BCYRN1 and miR-204-5p. MiR-204-5p has been confirmed to function as tumor suppressor in GC [10–16]. Therefore, we tried to explore the relationship between BCYRN1 and miR-204-5p in regulating GC cell proliferation, cell cycle, migration and invasion.

## Materials and methods

### Clinical specimens

A total of fresh 127 GC tissue samples and 35 paired non-tumor tissue samples were collected from patients who underwent surgical resection or biopsy at Xianyang Central Hospital or Yanan University Affiliated Hospital. All clinical specimens were confirmed by pathologists, and stored under liquid nitrogen until use. None of the GC patients received any anti-tumor therapy prior to pathologic diagnosis. The study was approved by the Ethics Committee of Xianyang Central Hospital and Yanan University Affiliated Hospital. All experiments were conducted in compliance with government policies and the Helsinki Declaration. The informed consent was obtained from each patient.

### Quantitative real-time polymerase chain reaction

Total RNAs were extracted and isolated from tissues and cells by TRIzol reagent (Invitrogen, Carlsbad, CA, U.S.A.) according to the manufacturer’s protocol. For detecting BCYRN1 expression, the PrimeScript RT Master Mix (Takara Biomedical Technology, Beijing, China) was used to synthesize complementary DNA, and One Step TB Green PrimeScript RT-PCR Kit (Takara Biomedical Technology, Beijing, China) was utilized to conduct quantitative real-time polymerase chain reaction (qRT-PCR) analysis in 7500 Real-Time PCR System (Applied Biosystems, Waltham, MA, U.S.A.). For detecting miR-204-5p expression, the Mir-X miRNA First Strand Synthesis Kit (Takara Biomedical Technology, Beijing, China) was utilized to synthesize complementary DNA, and Mir-X miRNA qRT-PCR TB Green Kit (Takara Biomedical Technology, Beijing, China) was applied to perform qRT-PCR analysis. U6 and GAPDH served as endogenous controls.

### Cell culture and transfection

Two GC cell lines BGC-823 and AGS, and a human gastric epithelium cell line GES-1 (Carlsbad, CA, U.S.A.) were cultured in RPMI-1640 medium (Gibco, Carlsbad, CA, U.S.A.) supplemented with 10% fetal bovine serum (FBS, Gibco, Carlsbad, CA, U.S.A.) in humidified air with 5% carbon dioxide and 37°C.

siRNA targeting BCYRN1 (si-BCYRN1), negative control siRNA (si-NC), miR-204-5p mimic, negative control mimic (mimics-NC), miR-204-5p inhibitor and negative control inhibitor (inhibitor-NC) were designed and synthesized by RiboBio Co., Ltd (Guangzhou, China). Lipofectamine 3000 reagent (Invitrogen, Carlsbad, CA, U.S.A.) was used for cell transfection in accordance with the manufacturer’s protocol.

### Luciferase reporter assay

The fragments of BCYRN1 containing miR-204-5p binding sites was amplified by PCR and cloned into the pmirGLO luciferase vectors (Promega, Madison, WI, U.S.A.), and named as wt-BCYRN1 and mut-BCYRN1, respectively. Then, GC cells were cotransfected with wt-BCYRN1/mut-BCYRN1 and miR-204-5p mimic/miR-204-5p inhibitor through Lipofectamine 3000 reagent. After 48 h, GC cells were collected and the Dual-Luciferase Reporter Assay System (Promega, Madison, WI, U.S.A.) was used to detect the luciferase activity.

### Cell count kit-8 assay

Cell viability was estimated by using Cell count kit-8 (CCK-8) assay at 24, 72, and 120 h after transfection. GC cells (2 × 10^4^) were seeded in 96-well plates, and were added with 10 μl CCK-8 solution (Dojindo Molecular Technologies, Kumamoto, Japan) at the indicated time. Then, GC cells were incubated at 37°C for 2 h, and the absorbance of the each well was detected using a microplate reader at a wavelength of 450 nm.

### Colony formation assay

The transfected GC cells were seeded into six-well plates at density of 400 cells per well and cultured for 14 days in humidified air with 5% carbon dioxide and 37°C. Then, the GC cells were fixed in methanol for 30 min and stained with Crystal Violet for 20 min. Colonies containing more than 50 cells were counted and compared.

### Cell-cycle analysis

The cell cycle of GC cells was analyzed using flow cytometric analysis. The transfected GC cells were collected, and fixed with 70% ethanol at 4°C overnight. Then cells were stained with 100 μl RNaseA and 400 μl Propidium Iodide for 40 min in the dark. Cell-cycle distribution was detected on the flow cytometry (FACScan, BD Biosciences, U.S.A.).

### Transwell cell migration and invasion assays

Transwell chambers were utilized to estimate cell migration and invasion abilities (Corning, Franklin Lakes, NJ, U.S.A.) with 8-μm pore size based on the manufacturer’s recommendations. For cell migration assay, 1 × 10^5^ GC cells in 200 μl serum-free RPMI-1640 medium were added into the upper chamber, and 500 μl RPMI-1640 medium containing 15% FBS was added into the lower chamber. After incubation for 24 h, GC cells resting on the upper filter were removed by a cotton swab, and GC cells migrating to the lower chamber were fixed by ethanol and stained using Crystal Violet. For invasion assay, all steps were the same with that in migration assay except that the upper chambers were pre-coated with Matrigel (BD Biosciences, San Jose, CA, U.S.A.). The number of migrated or invaded cells at five random fields is counted under a microscope.

### Statistical analysis

All statistical data were analyzed using SPSS 22.0 statistical software (IBM Corp., Armonk, NY, U.S.A.). All experiments were independently repeated three times. The Student’s *t* test was utilized for statistical comparison between two groups. Survival curve was estimated by Kaplan–Meier method and log-rank test. The univariate and multivariate Cox proportional hazards’ models were used for evaluating prognostic variables in GC patients. The correlation between BCYRN1 expression and miR-204-5p expression was assessed by Spearman’s correlation analysis. Associations between BCYRN1 expression and clinicopathologic characteristics of GC cases were estimated by Chi square test. *P*<0.05 was defined as a statistically significant difference.

## Results

### BCYRN1 is overexpressed in GC tissues and cell lines

At first, we analyzed the The Cancer Genome Atlas (TCGA) database to determine whether BCYRN1 is dysregulated in GC. We observed that BCYRN1 expression was obviously higher in GC tissues than in the adjacent normal tissues in TCGA database (*P*<0.001, Figure 1A). Furthermore, we performed qRT-PCR to confirm the expression of BCYRN1 between GC tissues and the adjacent normal tissues. We also found BCYRN1 was dramatically elevated in GC tissues compared with that in the adjacent normal tissues (*P*<0.001, Figure 1B). Then, the expression levels of BCYRN1 in GC cell lines and gastric epithelium cell line were also measured by qRT-PCR. The result revealed that BCYRN1 was notably overexpressed in GC cell lines compared with gastric epithelium cell line (*P*<0.001, Figure 1C). We induced down-regulation of BCYRN1 in GCs through siRNA transfection, and the transfection efficiency was confirmed by qRT-PCR (Figure 1D).

**Figure 1:** BCYRN1 is overexpressed in GC tissues and cell lines (**A**) BCYRN1 expression was higher in GC tissues than in the adjacent normal tissues in TCGA database. (**B**) BCYRN1 expression was higher in GC tissues than in the adjacent normal tissues in TCGA database. (**C**) BCYRN1 was overexpressed in GC cell lines compared with gastric epithelium cell line. (**D**) Down-regulation of BCYRN1 was induced in GCs through siRNA transfection (***P<0.001).

### BCYRN1 is associated with clinicopathological characteristics in GC patients

To further explore the clinical value of BCYRN1 in GC patients, we estimated the association between BCYRN1 expression and clinicopathological characteristics through Chi square test. First, all GC cases are divided into low BCYRN1 expression group and high BCYRN1 expression group based on the median value of BCYRN1 expression. As shown in Table 1, BCYRN1 expression was closely correlated with tumor depth (*P*=0.002), lymph node metastasis (*P*=0.001) and clinical stage (*P*<0.001) in patients with GC. However, BCYRN1 expression in GC patients had no association with gender (*P*=0.0324), age (*P*=0.774) and distant metastasis (*P*=0.138).

**Table 1:** Correlations between BCYRN1 expression and clinicopathological characteristics in GC

Characteristics	*n*	High expression	Low expression	*P*
Gender				
Female	47	26 (55.3)	21 (44.7)	0.324
Male	80	37 (46.3)	43 (53.8)	
Age (y)				
<50	52	25 (48.1)	27 (51.9)	0.774
≥50	75	38 (50.7)	37 (49.3)	
Clinical stage				
I-II	58	18 (31.0)	40 (69.0)	<0.001
III-IV	69	45 (65.2)	24 (34.8)	
Tumor depth				
T1-T2	64	23 (35.9)	41 (64.1)	0.002
T3-T4	63	40 (63.5)	23 (36.5)	
Lymph node metastasis				
N0-N1	65	22 (33.8)	43 (66.2)	0.001
N2-N3	62	41 (66.1)	21 (33.9)	
Distant metastasis				
M0	119	57 (47.9)	62 (52.1)	0.138
M1	8	6 (75.0)	2 (25.0)	

### BCYRN1 overexpression predicts an unfavorable prognosis in GC patients

To study the prognostic significance of BCYRN1 in GC patients, we evaluated the association between BCYRN1 expression and overall survival through Kaplan–Meier method and log-rank test. As presented in Figure 2, GC patients with high expression of BCYRN1 had worse overall survival in comparison with those with low expression of BCYRN1 (*P*<0.001). Furthermore, univariate and multivariate Cox regression analyses demonstrated that BCYRN1 expression (*P*=0.010, Table 2), tumor depth (*P*=0.026, Table 2) and distant metastasis (*P*<0.001, Table 2) were independent prognostic factors for overall survival in GC patients.

**Figure 2:** BCYRN1 overexpression predicts an unfavorable prognosis in GC patients The association between BCYRN1 expression and overall survival was estimated through Kaplan–Meier method and log-rank test.

**Table 2:** Univariate and multivariate Cox regression analyses of overall survival in GC patients

Parameter	Univariate analysis			Multivariate analysis		
	HR	95% CI	*P*	HR	95% CI	*P*
Gender						
(Male vs. Female)	0.875	0.549–1.392	0.572			
Age						
(≥50 vs. <50)	1.158	0.730–1.837	0.533			
Clinical stage						
(III-IV vs. I-II)	4.524	2.635–7.770	<0.001	2.978	0.876–10.126	0.081
Tumor depth						
(T3-T4 vs. T1-T2)	2.109	1.323–3.362	0.002	1.773	1.072–2.932	0.026
Lymph node metastasis						
(N2-N3 vs. N0-N1)	4.233	2.500–7.167	<0.001	1.120	0.328–3.824	0.856
Distant metastasis						
(M1 vs. M0)	13.301	5.256–33.656	<0.001	8.535	3.034–24.009	<0.001
BCYRN1						
(Low vs. High)	3.125	1942–5.030	<0.001	2.047	1.185–3.534	0.010

Abbreviations: HR, hazard ratio; 95% CI, 95% confidence interval.

### The relationship between BCYRN1 and miR-204-5p in GC

In LncBase predicted v.2 of DIANA tools, we found miR-204-5p was the predicted target of BCYRN1 (Figure 3A). In addition, we observed that there was a negative correlation between BCYRN1 and miR-204-5p in GC tissues (r = −0.624, *P*<0.001, Figure 3B). For exploring the relationship between miR-204-5p and BCYRN1, we conducted the luciferase reporter assay. Our data showed transfection of miR-204-5p mimics obviously decreased the luciferase activity of wt-BCYRN1 (*P*<0.001, Figure 3C) whereas miR-204-5p inhibitor dramatically increases the luciferase activity of wt-BCYRN1 in GC cells (*P*<0.001, Figure 3C), which indicated that BCYRN1 was directly bound to miR-204-5p. Then, we explored the effect of BCYRN1 on miR-204-5p expression in GC cells, and found knockdown of BCYRN1 expression significantly decreased miR-204-5p expression in GC cells (*P*<0.01, Figure 3D).

**Figure 3:** The relationship between BCYRN1 and miR-204-5p in GC (**A**) There were putative binding sites between BCYRN1 and miR-204-5p in lncRNA-microRNA interactome database. (**B**) There was a negative correlation between BCYRN1 and miR-204-5p in GC tissues. (**C**) Luciferase reporter assay showed that BCYRN1 directly bound to miR-204-5p. (**D**) Knockdown of BCYRN1 expression was significantly decreased miR-204-5p expression in GC cells (**P<0.01;***P<0.001).

### BCYRN1 regulates GC cell proliferation, cell cycle, migration and invasion through miR-204-5p

The published study suggested down-regulation of BCYRN1 inhibited GC cell proliferation, migration and invasion *in vitro* [9]. The growth curves and colony formation assay showed that down-regulation of BCYRN1 obviously suppressed GC cell proliferation (*P*<0.001, Figure 4A; *P*<0.05, Figure 4B). Furthermore, we observed that down-regulation of BCYRN1 blocked cell cycle transition from G_1_ to S and G_2_ phases (*P*<0.05, Figure 4C). Moreover, the transwell cell migration and invasion assays showed down-regulation of BCYRN1 inhibited GC cell migration and invasion (*P*<0.001, Figure 4D,E). In addition, we co-transfected si-BCYRN1 and miR-204-5p mimics/miR-204-5p inhibitor into GC cells to find out whether BCYRN1 affects the biological processes of GC cells via modulating miR-204-5p. As presented in Figure 4, miR-204-5p mimics reversed the obvious reduction by down-regulation of BCYRN1 on GC cell proliferation (*P*<0.001, Figure 4A; *P*<0.05, Figure 4B), cell-cycle arrest (*P*<0.05, Figure 4C), migration (*P*<0.001, Figure 4D) and invasion (*P*<0.001, Figure 4E). Moreover, miR-204-5p inhibitor did not further enhance the inhibitory effects of down-regulation of BCYRN1 on GC cell proliferation (*P*>0.05, Figure 4A,B), cell-cycle arrest (*P*>0.05, Figure 4C), migration (*P*>0.05, Figure 4D) and invasion (*P*>0.05, Figure 4E).

**Figure 4:** BCYRN1 regulates GC cell proliferation, cell-cycle, migration and invasion through miR-204-5p (**A**) The effect of BCYRN1 and miR-204-5p on GC cell viability was estimated by CCK-8 assay. (**B**) The effect of BCYRN1 and miR-204-5p on GC cell proliferation was evaluated by clone formation assay. (**C**) The effect of BCYRN1 and miR-204-5p on GC cell-cycle was analyzed by flow cytometry. (**D**) The effect of BCYRN1 and miR-204-5p on GC cell migration was detected by Transwell cell migration assay. (**E**) The effect of BCYRN1 and miR-204-5p on GC cell invasion was assessed by Transwell cell invasion assay (*P<0.05; ***P<0.001; Δ*P*>0.05).

## Discussion

BCYRN1 is a 200-nucleotide ncRNA originally identified as a neuron-specific transcript [17]. Recently, increasing studies showed that BCYRN1 is abnormally overexpressed in various types of human tumor tissues such as lung cancer [18,19], breast cancer [20,21], esophageal squamous cell carcinoma [22], colorectal cancer [23], cervical cancer [24] and glioma [25]. In GC, Ren et al. [9] found BCYRN1 expression in primary GC tissue sample and cell lines compared with their paired adjacent normal gastric tissue normal gastric epithelial cell line, respectively. Moreover, Lu et al. [26] suggested early GC tissues had significantly increased BCYRN1 expression in comparison with normal adjacent tissues, and BCYRN1 expression had potential diagnostic value (AUC = 0.821; sensitivity = 67.9%; specificity = 85.9%). However, there was a weak positive correlation observed between early GC tissues and plasma for BCYRN1 expression [26]. In our study, we observed that BCYRN1 expression was obviously higher in GC tissues than in the adjacent normal tissues at TCGA database. Then, we confirmed BCYRN1 was overexpressed in GC tissues and cell lines, which is consistent with above studies. However, Wu et al. [27] found BCYRN1 expression was markedly decreased in ovarian cancer samples compared with normal ovarian samples.

To further explore the clinical value of BCYRN1 in GC patients, we estimated the association between BCYRN1 expression and clinicopathological characteristics, and found that BCYRN1 expression was closely correlated with tumor depth, lymph node metastasis and clinical stage in patients with GC. Likewise, Ren et al. [9] suggested BCYRN1 overexpression was associated with advanced TNM stage and large tumor size in GC cases. However, no remarkable association was identified between BCYRN1 expression and clinicopathological characteristics of GC patients [26]. Besides, Gu et al. and Wu et al. [23,28] conformably demonstrated that high BCYRN1 expression was correlated with later TNM stage and longer tumor diameter in patients with GC. In breast cancer patients, levels of BCYRN1 expression were significantly increased in patients with ER-positive expression [29].

Up to now, the prognostic value of BCYRN1 expression was investigated in esophageal squamous cell carcinoma [22], colorectal cancer [28] and lung cancer [30]. The relation between BCYRN1 expression and clinical outcome was still unknown in GC patients. In our study, we found GC patients with high expression of BCYRN1 had worse overall survival in comparison with those with low expression of BCYRN1. Meanwhile, we identified high BCYRN1 expression as an independent prognostic factor for overall survival in GC patients. Similarly, Zhao et al. [22] found high BCYRN1 expression was negatively associated with shorter disease-free survival and overall survival, and acted as an independent prognostic factor for disease-free survival and overall survival in paitents with esophageal squamous cell carcinoma. In colon cancer patients, Wu et al. [28] showed the cumulative overall survival rate was obviously reduced in patients with high expression of BCYRN1 than in the patients with low expression of BCYRN1. In addition, Gao et al. [30] indicated that BCYRN1 overexpression was obviously correlated with poor clinical outcome in patients with non-small cell lung cancer.

BCYRN1 has been found by Ren et al. [9] to function as an oncogenic lncRNA in regulating GC cell proliferation, migration and invasion. Interestingly, we analyzed lncRNA-microRNA interactome database, and found that there were putative binding sites between BCYRN1 and miR-204-5p. Furthermore, we confirmed that down-regulation of BCYRN1 inhibited GC cell proliferation, cell-cycle arrest, migration and invasion through directly up-regulated miR-204-5p expression. In non-small cell lung cancer, Hu and Lu [18] found c-MYC activated BCYRN1 to promote tumor cell metastasis through up-regulating MMP-9 and MMP-13 [28]. Besides, down-regulation of BCYRN1 suppressed cell proliferation, migration and invasion, enhanced cell apoptosis, and induced cell-cycle arrest at G_0_/G_1_ phase [23]. However, Wu et al. [27] suggested silencing of BCYRN1 enhanced cell proliferation and reduced the sensitivity of carboplatin in ovarian cancer. The discrepancy of Wu et al.’s [27] data in ovarian cancer would be most likely due to tumor heterogenicity.

In conclusion, high expression of BCYRN1 predicts clinical progression and unfavorable prognosis in GC patients. Down-regulation of BCYRN1 inhibited GC cell proliferation, cell-cycle arrest, migration and invasion through directly up-regulated miR-204-5p expression.

## Abbreviations

AUC: area under curve
BCYRN1: brain cytoplasmic RNA 1
CCK-8: cell count kit-8
ER: estrogen receptor
FBS: fetal bovine serum
GC: gastric cancer
ncRNA: non-coding RNA
qRT-PCR: quantitative real-time polymerase chain reaction
TCGA: The Cancer Genome Atlas
TNM: tumor, lymph node, metastasis

## References

[1] BrayF., FerlayJ., SoerjomataramI., SiegelR.L., TorreL.A.and JemalA. (2018) Global cancer statistics 2018: GLOBOCAN estimates of incidence and mortality worldwide for 36 cancers in 185 countries. CA Cancer J. Clin. 68, 394–424 10.3322/caac.2149230207593

[2] DuarteH.O., GomesJ., MachadoJ.C.and ReisC.A. (2018) Gastric cancer: basic aspects. Helicobacter 23, e1252310.1111/hel.1252330277636

[3] TanA.C., ChanD.L., FaisalW.and PavlakisN. (2018) New drug developments in metastatic gastric cancer. Therap. Adv. Gastroenterol. 11, 175628481880807210.1177/175628481880807230455742PMC6236851

[4] VeneritoM., VasapolliR., RokkasT.and MalfertheinerP. (2018) Gastric cancer: epidemiology, prevention, and therapy. Helicobacter 23, e1251810.1111/hel.1251830203589

[5] ShinH., KimY., KimM.and LeeY. (2018) BC200 RNA: an emerging therapeutic target and diagnostic marker for human cancer. Mol. Cells 41, 993–999 3059090610.14348/molcells.2018.0425PMC6315322

[6] LuoQ.and ChenY. (2016) Long noncoding RNAs and Alzheimer’s disease. Clin. Interv. Aging 11, 867–872 10.2147/CIA.S10703727418812PMC4933566

[7] WuP., ZuoX., DengH., LiuX., LiuL.and JiA. (2013) Roles of long noncoding RNAs in brain development, functional diversification and neurodegenerative diseases. Brain Res. Bull. 97, 69–80 10.1016/j.brainresbull.2013.06.00123756188

[8] SamsonJ., CroninS.and DeanK. (2018) BC200 (BCYRN1) - The shortest, long, non-coding RNA associated with cancer. Noncoding RNA Res. 3, 131–143 10.1016/j.ncrna.2018.05.00330175286PMC6114260

[9] RenH., YangX., YangY., ZhangX., ZhaoR., WeiR.et al. (2018) Upregulation of LncRNA BCYRN1 promotes tumor progression and enhances EpCAM expression in gastric carcinoma. Oncotarget 9, 4851–4861 10.18632/oncotarget.2358529435146PMC5797017

[10] ZhouX., LiL., SuJ.and ZhangG. (2014) Decreased miR-204 in H. pylori-associated gastric cancer promotes cancer cell proliferation and invasion by targeting SOX4. PLoS ONE 9, e10145710.1371/journal.pone.010145724984017PMC4077842

[11] ZhangL., WangX.and ChenP. (2013) MiR-204 down regulates SIRT1 and reverts SIRT1-induced epithelial-mesenchymal transition, anoikis resistance and invasion in gastric cancer cells. BMC Cancer 13, 29010.1186/1471-2407-13-29023768087PMC3710153

[12] ZhangB., YinY., HuY., ZhangJ., BianZ., SongM.et al. (2015) MicroRNA-204-5p inhibits gastric cancer cell proliferation by downregulating USP47 and RAB22A. Med. Oncol. 32, 33110.1007/s12032-014-0331-y25429829

[13] YangS., CuiJ., YangY., LiuZ., YanH., TangC.et al. (2016) Over-expressed RPL34 promotes malignant proliferation of non-small cell lung cancer cells. Gene 576, 421–428 10.1016/j.gene.2015.10.05326526135

[14] ChenX., LiuX.S., LiuH.Y., LuY.Y.and LiY. (2016) Reduced expression of serum miR-204 predicts poor prognosis of gastric cancer. Genet. Mol. Res. 15, gmr770210.4238/gmr.1502770227173244

[15] YuanX., WangS., LiuM., LuZ., ZhanY., WangW.et al. (2017) Histological and pathological assessment of miR-204 and SOX4 levels in gastric cancer patients. Biomed. Res. Int. 2017, 689467510.1155/2017/689467528133610PMC5241485

[16] ShresthaS., YangC.D., HongH.C., ChouC.H., TaiC.S., ChiewM.Y.et al. (2017) Integrated MicroRNA-mRNA analysis reveals miR-204 inhibits cell proliferation in gastric cancer by targeting CKS1B, CXCL1 and GPRC5A. Int. J. Mol. Sci. 19, Pii: E8710.3390/ijms1901008729283424PMC5796037

[17] SosinskaP., Mikula-PietrasikJ.and KsiazekK. (2015) The double-edged sword of long non-coding RNA: The role of human brain-specific BC200 RNA in translational control, neurodegenerative diseases, and cancer. Mutat. Res. Rev. Mutat. Res. 766, 58–67 10.1016/j.mrrev.2015.08.00226596549

[18] HuT.and LuY.R. (2015) BCYRN1, a c-MYC-activated long non-coding RNA, regulates cell metastasis of non-small-cell lung cancer. Cancer Cell Int. 15, 3610.1186/s12935-015-0183-325866480PMC4392634

[19] WangY., BaiW., WangM., YuT.and ZhangW. (2019) Long non-coding RNA brain cytoplasmic RNA 1 acts as an oncogene and regulates cell proliferation and metastasis in non-small cell lung cancer. J. Nanosci. Nanotechnol. 19, 1978–1985 10.1166/jnn.2019.1640230486938

[20] IacoangeliA., AdzovicL., ChenE.Q., Latif CattieR., SoffG.A.and TiedgeH. (2018) Regulatory BC200 RNA in peripheral blood of patients with invasive breast cancer. J. Investig. Med. 66, 1055–1063 10.1136/jim-2018-00071729967012PMC6158080

[21] IacoangeliA., LinY., MorleyE.J., MuslimovI.A., BianchiR., ReillyJ.et al. (2004) BC200 RNA in invasive and preinvasive breast cancer. Carcinogenesis 25, 2125–2133 10.1093/carcin/bgh22815240511

[22] ZhaoR.H., ZhuC.H., LiX.K., CaoW., ZongH., CaoX.G.et al. (2016) BC200 LncRNA a potential predictive marker of poor prognosis in esophageal squamous cell carcinoma patients. Onco Targets Ther. 9, 2221–2226 2714391710.2147/OTT.S99401PMC4846077

[23] GuL., LuL., ZhouD.and LiuZ. (2018) Long noncoding RNA BCYRN1 promotes the proliferation of colorectal cancer cells via up-regulating NPR3 expression. Cell. Physiol. Biochem. 48, 2337–2349 10.1159/00049264930114690

[24] PengJ., HouF., FengJ., XuS.X.and MengX.Y. (2018) Long non-coding RNA BCYRN1 promotes the proliferation and metastasis of cervical cancer via targeting microRNA-138 *in vitro* and *in vivo*. Oncol. Lett. 15, 5809–5818 2955221210.3892/ol.2018.8015PMC5840573

[25] KrausT.F., GreinerA., GuibourtV., LisecK.and KretzschmarH.A. (2015) Identification of stably expressed lncRNAs as valid endogenous controls for profiling of human glioma. J. Cancer 6, 111–119 10.7150/jca.1086725561975PMC4280393

[26] LuQ., YuT., OuX., CaoD., XieT.and ChenX. (2017) Potential lncRNA diagnostic biomarkers for early gastric cancer. Mol. Med. Rep. 16, 9545–9552 10.3892/mmr.2017.777029039538

[27] WuD.I., WangT., RenC., LiuL., KongD., JinX.et al. (2016) Downregulation of BC200 in ovarian cancer contributes to cancer cell proliferation and chemoresistance to carboplatin. Oncol. Lett. 11, 1189–1194 10.3892/ol.2015.398326893717PMC4734031

[28] WuK., XuK., LiuK., HuangJ., ChenJ., ZhangJ.et al. (2018) Long noncoding RNA BC200 regulates cell growth and invasion in colon cancer. Int. J. Biochem. Cell Biol. 99, 219–225 10.1016/j.biocel.2018.04.00129625226

[29] SinghR., GuptaS.C., PengW.X., ZhouN., PochampallyR., AtfiA.et al. (2016) Regulation of alternative splicing of Bcl-x by BC200 contributes to breast cancer pathogenesis. Cell Death Dis. 7, e226210.1038/cddis.2016.16827277684PMC5143396

[30] GaoB.B.and WangS.X. (2019) LncRNA BC200 regulates the cell proliferation and cisplatin resistance in non-small cell lung cancer via PI3K/AKT pathway. Eur. Rev. Med. Pharmacol. Sci. 23, 1093–1101 3077907710.26355/eurrev_201902_16999

